The article "Enhancement of Nursing Effect in Emergency General Surgery Based on Computer Aid" was published in 2022. Journal: J Healthc Eng.

# Enhancement of Nursing Effect in Emergency General Surgery Based on Computer Aid

**DOI:** 10.1155/2022/6745993

**Published:** 2022-03-10

**Authors:** Yan Lei, Linxiang He, Houqiang Huang

**Affiliations:** ^1^Department of Emergency, Anqing First People's Hospital of Anhui Medical University, Anqing, Anhui 246003, China; ^2^Department of Nursing, The Affiliated Hospital of Southwest Medical University, Luzhou, Sichuan 030699, China

## Abstract

In order to improve the nursing effect of emergency general surgery, this paper combines computer algorithms to carry out the intelligent management of general surgery nursing, and realizes the standardization of nursing information, the electronic nursing file, the precision of nursing workload, and the intelligentization of nursing quality control by means of informatization. This truly and objectively reflects the nursing operation and treatment situation, prevents the occurrence of some adverse events, and effectively reduces the workload of nursing care. Moreover, this paper uses a standardized software design method to define the software concept, and then conducts a detailed demand analysis of the nursing display function through detailed investigation, class work, discussion and analysis, and comparison decision-making methods. In addition, this paper compiles the software through strict coding standards, and finally designs test cases to test and improve the software. Through actual case studies, it can be seen that the computer-assisted emergency general surgery nursing method proposed in this paper has a certain progress compared with the traditional nursing method.

## 1. Introduction

The pre-examination and triage of emergency general surgery is relatively mature abroad. A large number of studies have proved the effectiveness and practicability of their respective triage standards, and the corresponding emergency triage process and path have been established for clinical use. The establishment of modern triage standards began in the 1990s [1]. Countries such as the United States, Australia, France, Canada, and the United Kingdom have successively established unified and standardized emergency triage procedures and standards.

These triage standards are all five-level triage, and patients are divided into five levels according to the degree of criticality, of which level I is the most critical and urgent patient, and level V is the mildest nonemergency patient. Regarding the evaluation of the American ESI standard, there are still some studies that indicate that the triage standard is not perfect. Although it is based on the allocation of emergency resources, it still has shortcomings [2]. First of all, the sensitivity of distinguishing between various levels of the disease is low. Almost half of the patients are classified as Class III patients according to the allocation of emergency resources [3]. This makes it difficult to identify truly potentially critical patients and get corresponding and adequate dynamic observations. Secondly, the standard does not have sufficient research conclusions to prove the correlation between the outcome of the disease after triage and the time of triage. Finally, the completion of triage is still based on subjective triage. From factors such as lack of clinical experience, human triage errors, and system defects to triage staff's errors in the initial clinical assessment (i.e., triage), it leads to serious consequences such as misdiagnosis, delayed treatment, unreasonable use of medical resources, and increased medical costs.

Computer information technology gradually began to be applied to hospital management in the form of a single computer. In the early 1990s, hospitals began to introduce computer health information systems (HIS). The creation and adoption of clinical decision support (CDS) system tools have changed the way medical professionals traditionally manage patient health, disease data, healthcare records, and diagnosis and treatment plans [4]. Preliminary studies have shown that this type of medical guidance may play an important role in patient management and triage, especially in clinical areas such as EDs [5]. The United States and Canada took the lead in introducing information applications into emergency triage. With the development of the Internet of Things technology, some scientific research institutions have developed what is called a wireless network disaster medical emergency response information system; electronic LED lights are used as patient triage labels, which replace traditional paper labels. In addition to comprehensive triage information, the general surgery nursing system adds critical value alarms, scope and effectiveness checks (such as allergy tests), and complex decision support (such as pregnancy calculators, ESI, etc.) compared with other triage software. Foreign information-based emergency triage decision-making tools continue to increase; scholars have begun to pay attention to the “high efficiency” brought about by information technology; the reliability and effectiveness of triage have also become a research hotspot. At the same time, triage tools are not only developed in information, but intelligent functions are gradually being designed and developed. The triage staff uses electronic shunt sensors to wirelessly collect the patient's life status, remotely monitor the patient's vital signs, and can be based on the classification. The patient location tracking provided by the diagnosis tag allows for triage.

In order to improve the nursing effect of emergency general surgery, this paper combines computer algorithms to carry out the intelligent management of general surgery nursing so as to improve the nursing effect of general surgery and provide a reference for the further improvement of the quality of follow-up general surgery nursing service.

## 2. Related Work

In the early 1970s, hospitals in the United States, Japan, and other hospitals began to try to apply large-scale commercial computers to hospital management, began to research and develop hospital information systems, and established HIS system prototypes. By the mid-1980s, nursing information systems began to be used in some large hospitals in developed countries. With the development and maturity of various new network information technologies, foreign nursing-related information systems have been relatively complete. With the strengthening of the degree of integration of hospital nursing information and hospital management systems, all aspects of hospital nursing can be effectively managed, and the safety of nursing behavior is protected to a certain extent [6]. The earliest application of computer systems to hospital management in China began in the early 1980s. However, due to technical limitations, it was mainly used in stand-alone applications at that time, such as outpatient systems, charging systems, material management systems, financial systems, and so on. In the mid-1990s, due to the development of local area networks and other technologies, the nursing information system under the wired local area network environment also began to be applied [7]. In the late 1990s, with the maturity of network technology, the process of hospital informatization began to accelerate in China. In particular, after entering the 21st century, hospital information construction began to keep up with the pace of international development, and began to establish a digital hospital with clinical information as the core, including the establishment of doctor workstations and nurse workstations [8]. In recent years, with the wave of mobile IT sweeping the world, the traditional medical IT field is also undergoing rapid changes. The application of barcode recognition, sensor control, wireless applications, and other technologies in the nursing field has greatly liberated the labor force, improving accuracy and efficiency. With the help of these new technologies [9], new breakthroughs have emerged in the development of nurses' work. Moreover, many nursing management concepts and ideas have ushered in the soil of application and blossomed. For example, the overall responsibility system of nursing system combined with the application of mobile nursing technology solves the ambiguity and simple one-sided problems of traditional functional nursing and improves nursing safety [10].

In general, the nursing system is developing rapidly toward specialization, mobility, and diversification. The nursing system has evolved from a single, submodule subordinate to HIS to an integrated mobile nursing system, that includes traditional nurse workstations, nursing medical records, nursing management, and nursing care. Specialized clinical nursing information systems are being developed for planning and nursing tasks [11]. Foreign nursing information systems started earlier and gradually developed and improved. They can integrate all electronic records generated during patient care into an organic whole, and can collect, store, and process patient execution information and nursing staff-related information. Forming a closed loop of medical order and nursing quality control [12], combined with clinical medicine and nursing professional knowledge, can analyze and research patient data, medical order data, and nursing data, which is a better quality service for patients in the treatment process. At present, most domestic hospitals have implemented inpatient nurse workstations, and some of the more advanced hospitals have implemented overall nursing information systems (including intensive care nursing systems, nursing knowledge bases, nursing plans, and mobile nurse workstations) [13].

With the continuous improvement of the level of nursing specialization, it has also promoted the development of nursing specialties. Since the introduction of the modified early warning score (MEWS) system in the United Kingdom, the observation and early warning of critically ill patients in nursing work have played a very important role [14]. The MEWS scoring method is a very simple system for evaluating the patient's condition and prognosis. It scores comprehensively according to the patient's objective indicators, such as body temperature, heart rate, respiratory rate, systolic blood pressure, and consciousness, so that the patient's critical condition can be scored to achieve the advantages of being scientific, fast, simple, and predicting the risk of the disease [15]. At present, the MEWS scoring method has been widely used in ICUs and the emergency department as a tool to assess the severity or potential risk of the disease, and provide certain early warning support for early detection, early treatment, and early rescue of critically ill patients [16], but it has not been promoted in the surgical ward. At the same time, because young nurses now account for a large proportion of the department, relatively speaking, the identification and attention to the condition of some critically ill patients has been weakened to a certain extent [17]. Nowadays, with the continuous improvement of people's living standards and the advent of an aging society, more and more general surgery patients are showing a trend of aging. However, the elderly have more basic diseases, more comorbidities, and rapid changes in their conditions. Therefore, the relevant data of the improved MEWS score table [18] is now being applied to general surgery wards, which has a positive significance for the early detection of patient condition changes and intervention, effectively improving nurses' awareness and warning of potentially critically ill patients and preventing accidents.

## 3. Computer-Aided Emergency General Surgery Nursing System

The hospital's intelligent nursing display system is a business system that applies and serves the internal use of the Arab League Central Hospital. At the same time, the hospital also uses the intelligent nursing display system as an important means and tool to promote the improvement of nursing management. From the perspective of the development of medical informatization, the construction of nursing informatization is gradually developing toward mobile, intelligent, and wearable models. The mobile nursing information system uses mobile devices such as tablet computers, PDAs, smart phones, and other portable mobile devices to collect and distribute data. It also includes the use of large-screen display devices for data display and push. This can effectively help medical staff to grasp patient diagnosis and treatment information in a dynamic, comprehensive, and timely manner, scientifically arrange and execute diagnosis and treatment and nursing plans so as to solve the query, and enter vital signs data and medical care data by medical staff anytime and anywhere. Moreover, it helps hospitals realize a patient-centered service concept and a quality-centered management model. The development of the hospital's intelligent nursing display system can enable nurses to perform medical behaviors in clinical nursing work, such as fluid infusion, physical sign collection, intake and output, treatment execution, daily care, etc., to follow the patient to complete the collection work at the bedside. Moreover, the application of mobile nursing information technology rationally optimizes the original work flow, thereby improving the efficiency and the quality of nursing work, meeting the management requirements of high-quality nursing, and handling various emergencies (such as crisis values) in a timely and accurate manner.

(1) Comprehensive nursing information integration: It connects various business application systems in the hospital through the hospital data integration platform. Moreover, it integrates multiple systems such as clinical nursing, nursing management, mobile nursing, intensive care, medical order system, inspection, cost accounting, and material management. In addition, it collects relevant data and incorporates it into the clinical data center to form a data warehouse for the main body of nursing information, which solves the problems of repeated data entry and data inconsistency in multiple systems, and displays it on demand after processing. (2) Automatic generation of nursing plan: It is a predefined nursing plan knowledge base, and intelligently formulates nursing plans based on doctors' orders, nursing evaluation results, special physical signs, and patient conditions, and displays the patient's nursing plan dynamically in real time with a graphical interface. (3) Intelligent reminder of emergencies: The system can remind various problems in nursing work in real time, and intelligently, such as drug allergy and drug contraindications, and promptly remind emergency events such as crisis value to avoid medical errors. (4) Multi-level information display: The system can use electronic whiteboards, handheld terminals, tablet computers, electronic large screens, and other intelligent terminal devices to display corresponding information to doctors, responsible nurses, head nurses, and nursing department managers as needed to meet the information needs of people at different levels.

The hospital's intelligent nursing display system should combine the development needs of the hospital's clinical business, adhere to the demand-led approach, refer to the best practices of domestic and foreign industry informatization, and explore the informatization development model with low cost, good results, and outstanding highlights. It is necessary to gradually promote the hospital's information planning and construction in clinical diagnosis and treatment, medical quality control, operation management, decision analysis and other related aspects, and introduce scientific, professional, and refined management methods and means to drive the hospital's management innovation and service innovation. At the same time, it is necessary to realize the standardization of the management process, the networking of work communication, the electronicization of documents and materials, the sharing of knowledge and experience, and the openness of public welfare information so as to realize the new work pattern of “orderly management, free communication, and perfect service” in the hospital. At present, nursing information management systems and mobile clinical information systems based on mobile nursing work, electronic nursing documents, and labeling of nursing items have been put into use in many large- and medium-sized hospitals in China. The hospital intelligent nursing display system is a part of the nursing system, and the overall goal of the system is to promote the improvement of the hospital's nursing quality capabilities. With the least participation of the nursing staff, it can provide the nursing staff with the greatest help, or assist the nursing staff to achieve the following functions: (1) It can realize the automatic check of drugs and patients to avoid medical errors; (2) it can greatly reduce the workload of nursing and reduce the work intensity of nurses; (3) it can improve the efficiency and quality of nursing, and improve the level of nursing service; (4) it standardizes the clinical medical care process and improves the hospital's clinical medical care management level; (5) it provides medical and nursing staff message reminders to provide faster nursing assistance for nursing work; (6) it realizes patient review and provides comparison of average admission data for nursing management; (7) it implements a high-quality nursing information technology support platform to ensure that medical staff can communicate with each other anytime and anywhere; (8) it establishes a fair assessment mechanism to increase the enthusiasm of nursing staff. In general, the construction of the hospital's intelligent nursing display system will bring brand-new changes to nursing work, optimize the nursing workflow, and provide patients with better nursing services.

The conceptual model design is actually the realization process of the conceptual model. The conceptual model is an abstraction of the real world, i.e., it artificially processes actual people, objects, things, and concepts, extracts the necessary characteristics needed to build the system, ignores some nonessential details, and accurately describes these characteristics with various concepts.

The above is a detailed description and research of each functional module in the community intelligent remote monitoring system. Based on the analysis and abstraction of system developers, end users, and customers, it is concluded that the community intelligent remote monitoring system should include six use cases including physiological parameter monitoring, alarm information processing, nursing, information query, information management, and data interface.  Figure 1 is the UML use case diagram of the system.

With reference to the above-detailed analysis of each use case of the system, we gradually refine the data objects of this part of the system, design a partial conceptual model, and determine the relationship between them. The partial conceptual model of the system is shown in Figure 2.

The partial conceptual model of the system is mainly composed of the client's basic information object, the client's relative information object, the doctor's information object, and the client's multi-physiological parameter object. The numbers on the relationship line indicate the corresponding relationship between the data objects. For example, there is a one-to-many relationship between basic customer information and multiple physiological parameter data, i.e., a customer object contains multiple physiological parameter information. Through the detailed design of the partial conceptual structure, the relationship between the data objects is truly reflected, and the foundation for the subsequent logical model design is laid.

The system hardware framework is shown in Figure 3 below. STM32 is used as the main processor, and the internal running program drives the Wi-Fi chip to send and receive data.

The driver framework of 88W8686 is shown in Figure 4 below, where the host driver (hereafter referred to as the Host Driver) is responsible for communicating with the firmware in 88W8686 (hereafter referred to as the Firmware), where Firmware is a program running in the Wi-Fi SoC chip. After the system is powered on, the processor downloads it to the Wi-Fi chip, and then the firmware can run in the SoC. Based on the ARM CPU, MAC, baseband module, radio frequency module, and hardware interface inside the SoC, functions such as hardware interface control, data service, 802.11 MAC layer management, and hardware control are implemented. There are two channels between the Host Driver and the Firmware: data channel and command channel. The data channel is used to transmit data to be sent and received, and the command channel is used to transmit control commands. The Host Driver sends the standard 802.3 frame to the WLAN Firmware in the SoC, and the WLAN Firmware processes it as an 802.11 frame and then sends it out wirelessly. After the WLAN Firmware receives the 802.11 frame, it converts it into an 802.3 frame, and then sends it to the Host Driver through the data channel.

## 4. Analysis of Nursing Effect in Emergency General Surgery Based on Computer Aid

We select the emergency general surgery inpatients admitted to the emergency department of this hospital from June 2019 to December 2020 as the research sample. According to the method of random allocation, they are divided into the experimental group and the control group. Among them, the control group used traditional general surgical nursing methods, and the experimental group used the intelligent computer-aided nursing system constructed in this paper. In addition, other intervention methods are the same. On this basis, we collect relevant data for comparative analysis.

  Risk management for patients: Medical staff need to strengthen the management of neurosurgery emergency, surgery, elderly and critical patients, and use bed guards for patients with inconvenient mobility to prevent patients from falling from beds and other injuries. Therefore, the floor should be kept dry, handrails should be added to the bathroom, related warning signs should be present in wet areas, and the wheels, brakes, and guardrails of the patient's bed should be checked regularly. The nurse's shift needs to be 15 minutes in advance, and the content of the shift at the bedside must be effectively verified. For patients with more serious illnesses, the nursing staff need to strengthen communication with their families and provide relevant psychological counseling.
  Risk management for nurses: It is necessary to strengthen professional training and risk management awareness of nurses so as to effectively improve the quality of nursing work. At the same time, it is also necessary to strengthen the communication skills of nurses to promote a more harmonious relationship between the doctors and the patients. Hospital units can regularly organize nurses to conduct neurosurgery technical training and theoretical learning so as to improve the proficiency of nurses in nursing operations. At the same time, it is also necessary to strengthen the nursing level, communication level, and drug use methods of the nursing staff to improve the quality of nursing work. In addition, it is necessary to organize nurses to conduct academic exchange meetings on a regular basis to realize the sharing of information resources. For nursing staff with low qualifications, guidance and supervision need to be strengthened.
  Environmental risk management: The environment of the nephrology ward needs to be kept clean and comfortable so as to create a comfortable and quiet atmosphere for patients to recuperate. It is necessary to effectively implement the ward visiting system to prevent patients from being disturbed in their recuperation. At the same time, the environment needs to be disinfected to prevent infections in patients.
  Risk management for the pipeline: Patients in the Department of Nephrology generally have more catheters indwelled, and the main purpose is to observe the patient's condition. Therefore, the catheter needs to be kept unobstructed, and a fixing device should be added to prevent the catheter from twisting and pulling. At the same time, it is also necessary to sterilize the pipelines to strengthen the operational hygiene awareness of the medical staff and prevent patients from becoming infected. In addition, the indwelling time of the catheter needs to be communicated with the physician to prevent infection caused by excessive indwelling time.
  Risk management for emergency treatment: It is necessary to carry out effective and reasonable treatment of emergency plans for intravenous extravasation of special drugs, emergency plans for blockages, emergency plans for pressure sore prevention, emergency plans for cross-infection, and emergency plans for power outages and water cuts. At the same time, it is necessary to carry out relevant emergency drills to improve the emergency awareness of nurses, strengthen the awareness and understanding of emergency handling, improve proficiency, and effectively guarantee the quality of emergency work. On this basis, the effects of computer-aided care in emergency general surgery are calculated, and the results are shown in Tables 1–4.

It can be seen from the above research that the computer-assisted emergency general surgery nursing method proposed in this paper has a certain progress compared with the traditional nursing method. Therefore, the system of this paper can be used as an auxiliary nursing system in the follow-up hospital emergency general surgery nursing to improve the nursing effect of emergency general surgery.

## 5. Conclusion

Emergency Department of General Surgery is a very important department, which is highly specialized and involves many types of diseases. In addition, the condition of some patients with craniocerebral trauma changes rapidly and the onset is more rapid; thus, medical personnel are more required to have skilled emergency handling capabilities and operational skills. The professional nature and the importance of the departments also determine the trend of nurses' high work intensity and workload. Under this highly stressful working state, the occurrence of medical care risks is also increasing. Therefore, nurses need to strengthen the analysis and management of risk factors in nursing work so as to prevent risk events. At the same time, hospital units also need to combine the items complained by patients and medical disputes, strengthen in-depth analysis and investigation of these events, understand and recognize the information content related to risk events, and evaluate the consequences of them so as to summarize the factors associated with risk events. In order to improve the nursing effect of emergency general surgery, this paper combines computer algorithms to carry out the intelligent management of general surgery nursing so as to improve the nursing effect of general surgery. Through actual case studies, it can be seen that the computer-assisted emergency general surgery nursing method proposed in this paper has a certain progress compared with the traditional nursing method.

## Figures and Tables

**Figure 1:** The use case diagram of a computer-aided emergency general surgery nursing system.

**Figure 2:** Partial conceptual model diagram.

**Figure 3:** Wi-Fi system hardware block diagram.

**Figure 4:** Hierarchical structure of the driver.

**Table 1:** The incidence of adverse nursing events in emergency general surgery.

No	Control group (%)	Test group (%)
1	8.65	1.85
2	7.19	1.95
3	4.59	0.69
4	5.53	0.18
5	4.52	1.21
6	4.37	1.94
7	4.12	1.12
8	3.85	1.16
9	8.60	0.86
10	6.48	1.15
11	6.66	0.23
12	2.32	0.44
13	4.88	0.55
14	8.64	0.70
15	6.38	1.46
16	4.96	0.87
17	4.33	1.91
18	4.18	0.18
19	5.36	1.19
20	5.37	0.71
21	8.27	0.59
22	7.43	0.55
23	1.99	0.67
24	1.76	0.82
25	8.89	0.95
26	4.13	0.09
27	2.48	0.92
28	1.23	0.50
29	8.93	1.03
30	3.68	0.69
31	4.88	1.44
32	2.81	0.02
33	4.49	1.83
34	5.21	0.19
35	6.80	0.95
36	2.48	1.93
37	1.65	1.08
38	1.75	0.30
39	3.84	1.96
40	7.04	0.39

**Table 2:** Completion rate of nursing measures in emergency general surgery.

No	Control group (%)	Test group (%)
1	91.62	97.63
2	93.00	97.41
3	90.16	97.55
4	91.71	95.28
5	87.09	98.68
6	85.70	94.09
7	90.84	97.15
8	93.92	94.28
9	91.50	99.73
10	92.53	99.86
11	92.20	98.95
12	91.87	99.17
13	93.63	94.09
14	87.97	94.17
15	89.87	95.64
16	93.03	98.29
17	87.92	96.48
18	92.55	98.97
19	87.01	94.80
20	90.12	98.38
21	87.74	95.22
22	91.66	95.60
23	88.53	97.18
24	85.45	97.62
25	91.95	99.01
26	92.94	98.35
27	93.08	96.24
28	91.15	97.40
29	91.17	96.33
30	92.75	98.01
31	86.31	95.10
32	93.32	97.56
33	90.18	99.63
34	86.24	94.79
35	91.82	95.74
36	89.92	99.89
37	91.85	96.86
38	92.30	98.03
39	86.73	96.78
40	85.82	98.97

**Table 3:** Satisfaction of nursing patients in emergency general surgery.

No	Control group	Test group
1	85.25	97.01
2	87.16	95.48
3	91.70	96.21
4	91.45	97.19
5	89.23	95.81
6	88.01	99.25
7	90.95	97.98
8	86.91	98.23
9	92.00	95.42
10	90.84	96.11
11	90.92	94.37
12	89.72	98.44
13	89.00	95.28
14	93.77	97.07
15	87.06	99.53
16	90.50	96.02
17	89.61	98.14
18	86.90	96.08
19	88.03	97.30
20	93.46	98.61
21	88.23	96.53
22	89.37	95.09
23	90.74	94.20
24	93.31	95.80
25	88.82	97.24
26	92.22	98.09
27	85.41	98.64
28	88.65	95.41
29	86.01	94.26
30	86.89	97.41
31	90.92	99.31
32	92.19	95.97
33	88.39	94.12
34	88.36	94.53
35	91.69	96.81
36	88.05	94.74
37	87.41	95.87
38	91.92	97.40
39	88.38	99.16
40	87.39	96.03

**Table 4:** Satisfaction of nursing doctors in emergency general surgery.

No	Control group	Test group
1	88.73	99.45
2	91.34	98.13
3	93.17	95.84
4	85.37	97.08
5	90.13	99.26
6	90.88	96.20
7	85.85	96.44
8	87.20	94.51
9	93.99	94.16
10	89.62	94.32
11	86.57	96.86
12	85.70	98.96
13	92.24	98.31
14	85.20	96.58
15	90.66	99.41
16	86.49	98.67
17	85.85	94.24
18	91.47	96.99
19	91.14	97.08
20	89.02	98.82
21	90.77	96.31
22	91.00	96.47
23	86.50	95.03
24	92.37	99.07
25	85.33	94.56
26	91.63	99.81
27	91.78	95.45
28	93.70	98.45
29	93.26	97.52
30	92.14	99.32
31	87.36	97.11
32	91.61	94.32
33	86.81	99.69
34	92.36	98.10
35	93.77	96.20
36	88.34	99.17
37	86.02	95.20
38	92.72	98.94
39	86.68	95.87
40	91.32	98.07

## Data Availability

The data used to support the findings of this study are available from the corresponding author upon request.
